# Transient Increase in Homocysteine but Not Hyperhomocysteinemia during Acute Exercise at Different Intensities in Sedentary Individuals

**DOI:** 10.1371/journal.pone.0051185

**Published:** 2012-12-07

**Authors:** Eduardo Iglesias-Gutiérrez, Brendan Egan, Ángel Enrique Díaz-Martínez, José Luis Peñalvo, Antonio González-Medina, Pablo Martínez-Camblor, Donal J. O’Gorman, Natalia Úbeda

**Affiliations:** 1 Department of Pharmaceutical and Food Sciences, CEU San Pablo University, Madrid, Spain; 2 Centre for Preventive Medicine, School of Health and Human Performance, Dublin City University, Dublin, Ireland; 3 Sports Medicine Center, Clinical Laboratory, Higher Council for Sports, Madrid, Spain; 4 Department of Cardiovascular Epidemiology and Population Genetics, National Center for Cardiovascular Research (CNIC), Madrid, Spain; 5 Biosanitary Research Office of Asturias, Foundation for Asturias Promotion of Applied Scientific Research and Technology (FICYT), Oviedo, Spain; Medical College of Georgia, United States of America

## Abstract

Considering that hyperhomocysteinemia is an independent risk factor for cardiovascular disease, the purpose of this study was to determine the kinetics of serum homocysteine (tHcy) and the vitamins involved in its metabolism (folates, B_12_, and B_6_) in response to acute exercise at different intensities. Eight sedentary males (18–27 yr) took part in the study. Subjects were required to complete two isocaloric (400 kcal) acute exercise trials on separate occasions at 40% (low intensity, LI) and 80% VO_2peak_ (high intensity, HI). Blood samples were drawn at different points before (pre4 and pre0 h), during (exer10, exer20, exer30, exer45, and exer60 min), and after exercise (post0, post3, and post19 h). Dietary, genetic, and lifestyle factors were controlled. Maximum tHcy occurred during exercise, both at LI (8.6 (8.0–10.1) µmol/L, 9.3% increase from pre0) and HI (9.4 (8.2–10.6) µmol/L, 25.7% increase from pre0), coinciding with an accumulated energy expenditure independent of the exercise intensity. From this point onwards tHcy declined until the cessation of exercise and continued descending. At post19, tHcy was not different from pre-exercise values. No values of hyperhomocysteinemia were observed at any sampling point and intensity. In conclusion, acute exercise in sedentary individuals, even at HI, shows no negative effect on tHcy when at least 400 kcal are spent during exercise and the nutritional status for folate, B_12_, and B_6_ is adequate, since no hyperhomocysteinemia has been observed and basal concentrations were recovered in less than 24 h. This could be relevant for further informing healthy exercise recommendations.

## Introduction

The response to exercise of risk factors for chronic and degenerative diseases needs to be fully characterized before exercise can be most effectively prescribed as a preventive tool [1]. Hyperhomocysteinemia has emerged as an independent risk factor for cardiovascular disease (CVD), via endothelial dysfunction, oxidative stress mechanisms and inflammatory vascular processes [2], [3], [4], [5]. It is well known that plasma homocysteine concentration (tHcy) is inversely associated with plasma concentrations of folate and vitamins B_12_ and B_6_ [6]. Furthermore, tHcy is strongly influenced by the intake of methionine, folate, vitamin B_12_, and vitamin B_6_, as well as by other dietary factors, such as animal protein, coffee and alcohol. Genetic predisposition, age, gender, medication use, and lifestyle factors such as smoking, also influence tHcy [7]. However, the impact of physical activity on tHcy remains unclear.

A lack of consensus exists based on previous studies, which appears to be related to heterogeneity in the experimental design and the lack of control of confounding variables [8], [9], [10]. Additionally, those studies that have analyzed the effect of an acute bout of exercise have examined tHcy only before and after exercise, and no information is available regarding the kinetics of tHcy during exercise.

Few articles have analyzed the effects of acute exercise on tHcy among sedentary individuals [11], [12], [13], despite the potential importance for public health of hyperhomocysteinemia and sedentarism. A recent survey on sport and physical activity in the European Union [14] reported that 60% of EU citizens either never play sport or only do so rarely (one to three times per month or less). Similarly, 34% of EU citizens affirm that they are either physically inactive or occasionally active [14]. Physical inactivity is considered an independent risk factor for CVD [15], [16], and acute aerobic exercise has been associated with transiently increasing CVD risk by inducing platelet aggregation and thrombosis [17]. Therefore, a large amount of sedentary people that seldom performs a single bout of exercise, could be at a higher CVD risk.

We hypothesized that tHcy would increase linearly in response to acute exercise in sedentary individuals, reaching values of hyperhomocysteinemia by the end of high intensity exercise. To test this hypothesis, we analyzed the complete tHcy kinetics in response to high and low intensity exercise in sedentary individuals, controlling dietary, genetic, and lifestyle factors. Surprisingly, our results revealed that, at both intensities, maximum tHcy occurred during exercise, coinciding with similar accumulated energy expenditure and no values of hyperhomocysteinemia were observed.

## Subjects and Methods

### Ethics Statement

All experimental procedures were approved by the Dublin City University Research Ethics Committee in accordance with the Declaration of Helsinki. All participants gave written informed consent.

### Experimental Design

In a randomized crossover design, subjects were required to complete two isocaloric acute exercise trials, consisting of cycle exercise at 40% (low intensity, LI) and 80% (high intensity, HI) VO_2peak_, in random order separated by at least one week. Seven days before the first experimental trial, the power outputs required to elicit 40% and 80% VO_2peak_ were verified. Each exercise bout required the participants to expend 400 kcal, determined by indirect calorimetry monitored on a minute-by-minute basis [18]. It has been suggested that the intensity of exercise should be adapted to allow a minimum expenditure of 300 kcal in each exercise session for developing and maintaining cardiorespiratory fitness [19]. The duration of both exercise trials was different as the relative energy expenditure in kcal·min^−1^ was different between trials reflecting the divergent exercise intensities, and thus a longer time was required to expend 400 kcal during LI (69.9±4.0 vs. 36.0±2.2 min, LI vs. HI respectively, P<0.01).

### Subjects

Participants were recruited using flyers posted on campus and e-mail sent to the student and staff mailing lists. Prior to participation, each volunteer underwent a thorough medical screening to determine eligibility. Eight young males (18–27 yr) who were healthy, non-obese and had been physically inactive for at least 6 months, took part in the study as previously described [20].

### Anthropometry and Aerobic Capacity Assessment

On their first visit, the participants had their body composition assessed and their peak oxygen uptake (VO_2peak_) determined at the Metabolic Physiology Research Unit.

Height and body mass (BM) were measured using a combined medical scale (model 778, Seca Ltd, Hamburgh, Germany; precision 0.1 cm for height and 0.1 kg for weight) and the body mass index (BMI) was calculated.

Body density was calculated by the method of Jackson & Pollock (1978) [21], based on the sum of seven skinfolds (triceps, subscapular, mid-axillary, pectoral, suprailiac, abdominal, thigh) measured with Harpenden skinfold calipers (Holtain Ltd., Crosswell, Crymych, Pembrokeshire, UK). Percentage body fat (%BF) was calculated using the equation of Siri (1961) [22].

VO_2peak_was determined by indirect calorimetry (Vmax 29C, SensorMedics, Yorba Linda, CA, USA) using an incremental protocol on an electronically braked stationary cycle ergometer (Ergoline 900, SensorMedics).

### Dietary Control

Participants were asked to keep a one-day food diary on the day prior to the first experimental trial and asked to repeat the content and pattern of dietary intake on the day preceding the second experimental trial. They were asked to abstain from caffeine and alcohol consumption for 24 h prior to testing, and none of them reported the use of vitamin supplements. Dietary records were analyzed using a nutrient analysis program (WISP, Tinuviel Software, UK) [23].

The dietary intake during each experimental trial was standardized in terms of food type and macronutrient composition, and individualized for each participant in terms of total energy content. The energy requirements were calculated using the Harris-Benedict equation [24], multiplied by a physical activity factor (1.4), and with 400 kcal added to account for the exercise trial [25]. Three meals, each with 30% of predicted total energy expenditure, were provided, with the remaining 10% energy supplied with an evening snack. In accordance with current Recommended Dietary Allowances (RDA) [26] and Acceptable Macronutrient Distribution Range (AMDR) [27], these meals were designed to provide 45–65%, 20–35%, and 10–35% of total energy intake from carbohydrate (CHO), fat and protein sources, respectively, as well as an adequate intake of folate, vitamin B_12_, and vitamin B_6_.

### Blood Sampling

For the experimental trials subjects reported to the laboratory after an overnight fast and had a blood sample taken (pre4). Subjects then consumed a standardized breakfast and remained in the laboratory for 4 h, at which point they started the exercise bout. Immediately before exercise another blood sample was taken (pre0). Participants began then cycling on a stationary ergometer (cadence at 70–75 rpm) and continued until 400 kcal were expended. During exercise blood samples were drawn every 10 min for the first 30 min (exer10, exer20, and exer30), and every 15 min thereafter (exer45 and exer60) until exhaustion, via catheter placed in the antecubital vein. Sampling points were the same for both exercise trials, although samples at exer45 and exer60 were only taken during LI due to its longer duration. The total volume of blood taken during the trial was less than 40 ml. Another blood sample was drawn immediately (post0) and 3 h after the cessation of exercise (post3). During this 3 h of recovery, subjects remained in the laboratory and were permitted to consume only water *ad libitum*. After the post3 blood sample, subjects were provided with a standard meal, after which consumption they were free to leave the laboratory. Another meal and snack were provided to eat later that evening, and water intake was permitted to their satisfaction. No other food or beverages were allowed. The following morning subjects returned to the laboratory at the same time as the previous day, after an overnight fast, for a final blood sample taken at 19 h after the cessation of exercise (post19).

The procedure was identical for both exercise trials with the exception of the exercise intensity and, therefore, the duration of the exercise bout.

Blood samples (4 ml) were collected in vacutainers (No Additive (Z), Becton Dickinson, Franklin Lakes, NJ), kept at room temperature for 20 min, and then centrifuged at 3000 rpm for 15 min at 4°C. The serum was stored at −80°C for later analysis.

### Biochemical Determinations

tHcy and serum vitamin B_6_ (Pyridoxal 5′-phosphate, PLP) were determined by HPLC using a commercially available kit (Chromsystems Instruments & Chemicals GmbH, Munich, Germany) and fluorescent detection, where a derivatization process of the sample takes place. Once the sample is prepared, 50 µl are injected into the HPLC and fluorescence is measured at 385 nm excitation and 515 nm emission for tHcy and at 370 nm excitation and 470 nm emission for vitamin B_6_.

Folate and vitamin B_12_ serum concentrations were measured using an ELECSYS system (Roche Diagnostics GmbH, D-68298 Mannheim, Germany) based on an electrochemiluminescence immunoassay (ECLIA).

### Genotyping

Subjects were genotyped for C677T methylene tetrahydrofolate reductase (MTHFR) polymorphism. DNA was extracted from a muscle biopsy taken in rested state from a routine procedure in a previous study [20]. A phenol:chloroform:isoamyl alcohol (25∶24∶1) extraction [28] was performed, followed by purification, achieved with Microcon-100 microconcentrators (Millipore, Billerica, MA) by following the manufacturer’s instructions.

Genotype analyses were done by PCR-restriction fragment-length polymorphism analysis and then separately cleaved with *Hinf*I restriction enzyme (Promega Corporation, Madison, WI). The restriction digest was analyzed by gel electrophoresis to identify each possible restriction fragment length polymorphism pattern characteristic of mutation as described by Frosst *et al*. (1995) [29].

### Statistical Analysis

Normality of variables was tested using Shapiro Wilk’s test. In light of the results obtained, descriptive values are presented as medians and interquartile range in parenthesis and non-parametric methods were used.

Results about the distribution of tHcy values at every sampling point during low and high intensity exercise are presented as grouped box plots.

Differences between medians were analyzed using Mann-Whithey *U* test for independent samples (comparisons between exercise intensities) and Friedman test followed by Wilcoxon test for related variables (comparisons between sampling points at the same intensity).

In order to check the relationship among the different variables at each time point, a full correlation analysis was made by using Pearson correlation coefficient on the respective logarithmic transformation.

The level of significance was set at p<0.05 for all analyses; for multiple testing, Bonferroni correction was considered. Descriptive and analytical statistical analyses were performed using IBM® SPSS® Statistics (version 19) (Somers, NY).

Characteristic kinetic parameters (Maximum concentration, Cmax and Time to maximum concentration, Tmax) of tHcy, folate, vitamin B_12_, and vitamin B_6_ in serum were assessed by noncompartmental residual technique resolving each obtained curve into a series of exponential terms corresponding to the absorption, distribution, and elimination phases of the compound assuming apparent first-order rate processes, evidenced by linearity in the terminal portion of a semi-log plot. The parameters were calculated with PK Solutions 2.0 Noncompartmental Pharmacokinetics Data Analysis software (Summit Research Services, Montrose, CO, USA).

## Results

Anthropometric characteristics (height, body mass, BMI, body fat) and aerobic capacity (VO_2peak_) of sedentary volunteers are shown in Table 1.

**Table 1:** Characteristics of the subjects (n = 8).

	Median	IR
Height (m)	1.79	(1.74–1.81)
Body mass (kg)	79.4	(74.2–87.3)
BMI (kg·m^−2^)	25.0	(21.5–28.4)
Sum of 7 skinfolds (mm)^a^	124.8	(56.4–184.9)
%BF^b^	17.0	(6.7–24.8)
VO_2peak_ (ml·kg^−1^·min^−1^)	38.0	(34.0–49.8)

a Sum of 7 skinfolds: triceps, pectoralis, subscapular, abdominal, mid-axilary, suprailliac, and thigh.

b Body density was calculated by the Jackson and Pollock (1978) equation [21] and %BF was estimated using the Siri (1961) equation [22].

IR: Interquartile range; %BF: Percentage of body fat; VO_2peak_: Peak oxygen uptake.

None of the individuals assessed was TT homozygote for C677T MTHFR polymorphism, while 75% (n = 6) were heterozygous (CT) and 25% were CC homozygotes.

Serum tHcy was not related to C677T MTHFR genotypes at any sampling point or exercise intensity.

The graphic representation of the serum clearance kinetics of tHcy, together with calculated Cmax and Tmax in response to LI and HI, are shown in Figure 1. Box plots (Figure 2) were used to represent the distribution of tHcy values at every sampling point during LI and HI.

**Figure 1:** Serum homocysteine kinetics and calculated Cmax and Tmax at low and high intensity isocaloric exercise trials. Solid line and black dots, Low intensity exercise (40% VO_2peak_); Dashed line and white dots, High intensity exercise (80% VO_2peak_). Data are presented as medians in the figure and medians (interquartile range) in the table. *Significant differences in high intensity exercise (*P*<0.05) between pre0 vs. exer10, exer20, exer30, and post0. †Significant differences in high intensity exercise (*P*<0.05) between post19 vs. exer10, 20, 30, post0, and post 3. LI: Low intensity exercise; HI: High intensity exercise; pre0: Blood sample immediately before exercise; exer10: Blood sample 10 min during exercise; exer20: Blood sample 20 min during exercise; exer30: Blood sample 30 min during exercise; post0: Blood sample immediately after exercise; post3: Blood sample 3 h after exercise; post19: Blood sample 19 h after exercise.

No statistical differences in tHcy were found at baseline (pre4 and pre0) between LI and HI (pre4∶8.1 (7.0–8.3) vs. 8.1 (7.2–10.0) µmol/L; pre0∶7.8 (7.0–8.3) vs. 7.4 (6.3–9.6) µmol/L).

A significant increase in tHcy was observed during HI, reaching Cmax after 25 min of exercise (9.4 (8.2–10.6) µmol/L). This represents 1.9 µmol/L higher than pre0 or a 25.7% increase. tHcy started decreasing progressively during the HI trial and continued after the cessation of exercise. At post19, tHcy was not different to baseline (LI, post19∶6.8 (6.3–8.2) µmol/L; HI, post19∶7.5 (6.8–8.2)). No values of hyperhomocysteinemia (tHcy>15 µmol/L) [5], [30] were observed at any sampling point.

tHcy response to LI was similar to that observed for HI and no statistically significant differences were observed between values obtained at the same sampling points in both trials. However, the increase observed in tHcy during LI was lower, reaching Cmax (8.6 (8.0–10.1) µmol/L) after 37.5 min of exercise, 0.8 µmol/L higher than pre0 or a 9.3% increase. No statistically significant differences were found between sampling points during LI exercise.

No statistically significant differences were found for Cmax at HI vs. LI exercise.

Although Cmax and Tmax for tHcy were different at LI and HI, no statistically significant differences were found for the energy expenditure at Cmax between both intensities (272.4 vs. 217.0 kcal, respectively).

Table 2 shows the serum concentration of folate, vitamin B_12_, and vitamin B_6_ at every sample point, together with calculated Cmax and Tmax in response to LI and HI. No statistical differences were found between LI and HI for serum folate, vitamin B_12_, and vitamin B_6_ concentrations neither at baseline nor at any other sampling point. The serum concentration of the three vitamins were adequate at every sampling point (folate: >3.4 nmol/L; vitamin B_12_: >120 pmol/L; vitamin B_6_: >30 nmol/L) [31].

**Table 2:** Serum folate, vitamin B_12_, and vitamin B_6_ concentration before, during, and after two acute isocaloric exercise trials at low and high intensity (LI, 40% VO_2peak_ and HI, 80% VO_2peak_) in sedentary volunteers (n = 8).

	Folate (nmol/L)		Vitamin B_12_ (pmol/L)		Vitamin B_6_ (pmol/L)	
	LI	HI	LI	HI	LI	HI
pre4	21.9 (15.1–32.1)*^a^*	20.5 (15.–30.9)*^b^*	412.2 (290.4–460.2)*^c^*	385.4 (295.2–511.2)	61.9 (36.8–137.3)*^f^*	52.5 (36.4–111.5)*^i^*
pre0	32.4 (16.0–38.8)	20.9 (13.7–39.6)	334.6 (246.8–438.2)*^d^*	349.4 (251.1–435.5)	119.5 (84.8–144.0)	94.3 (53.1–126.9)
exer10	25.1 (15.0–33.4)	26.0 (16.2–30.2)	299.8 (249.0–400.0)	343.2 (296.2–424.0)	139.4 (98.5–154.6)	105.2 (77.6–156.4)
exer20	29.9 (14.9–33.4)	23.7 (19.6–39.0)	340.6 (269.3–417.1)	368.5 (322.8–446.1)	169.7 (89.7–197.8)*^g^*	114.6 (59.9–155.3)
exer30	24.8 (14.9–37.8)	27.8 (16.8–38.3)	358.9 (280.1–428.1)	373.6 (321.6–461.8)	123.6 (92.4–175.1)	109.3 (68.8–172.8)
exer45	24.1 (15.9–44.4)	–	371.2 (290.8–430.5)	–	143.0 (85.9–202.0)	–
exer60	24.0 (15.8–55.2)	–	345.2 (243.4–427.9)	–	198.7 (81.7–218.6)	–
post0	26.3 (17.6–42.2)	25.6 (20.6–36.8)	422.2 (294.1–465.8)*^c^*	407.7 (327.0–434.4)*^e^*	135.8 (80.2–165.1)	104.1 (63.4–190.8)^j^
post3	24.3 (19.5–30.8)	21.3 (17.9–31.5)	423.2 (308.5–468.8)*^c^*	374.6 (297.5–399.4)	108.4 (84.6–135.9)	80.9 (52.9–154.0)
post19	21.7 (18.4–30.0)	21.7 (17.8–31.3)	418.6 (257.0–492.2)	363.2 (272.6–496.0)	92.8 (70.5–157.3)*^h^*	57.8 (39.6–137.4)*^k^*
Cmax	44.8 (17.6–62.6)	28.0 (21.8–41.9)	422.2 (328.5–449.4)	423.0 (328.5–449.4)	201.8 (125.6–218.9)	125.8 (81.2–193.4)
Tmax	50 (22–60)	20 (0–30)	55 (45–70)	30 (22–40)	25 (20–56)	25 (10–38)

Data are presented as Median (Interquartile range).

Significant difference (P<0.05) from: ^a^exer20, exer60, and post0; ^b^exer30; ^c^pre0, exer10, exer20, exer30, exer45, and exer60; ^d^post19; ^e^pre0, exer10, and post3; ^f^pre0, exer10, exer20, exer45, exer60, post0, and post3; ^g^post0, post3, and post19; ^h^from exer20, exer60, and post0; ^i^exer10, exer20, exer30, post0, and post3; ^j^pre4, pre0, post3, and post19; ^k^exer20, exer30, post0, and post3. HI: High intensity exercise; LI: Low intensity exercise; pre4: before exercise (4 h); pre0: immediately before exercise; exer10: during exercise (10 min); exer20: during exercise (20 min); exer30: during exercise (30 min); exer45: during exercise (45 min); exer60: during exercise (60 min); post0: immediately after exercise; post3: before exercise (3 h); post19: before exercise (19 h).

Serum folate concentration increased significantly during exercise. The increase was higher during LI compared to HI (Cmax: 44.8 nmol/L after 50 min vs. Cmax: 28.0 nmol/L after 20 min), although no significant differences were observed between trials. Folate concentration at post19 were not different from pre4, showing also a recovery from the baseline.

Vitamin B_12_ serum concentration decreased between pre4 and pre0 and during the first minutes of exercise, both for LI and HI. Then, its concentration increased continuously until the end of exercise, and serum concentration at post0 was significantly higher than at pre0 and exer10 for both intensities, reaching Cmax close to the end of exercise (LI: 422.2 pmol/L after 55 min; HI: 423.0 pmol/L after 30 min). Vitamin B_12_ concentration at post19 was not different from pre4.

Serum vitamin B_6_ concentration increased significantly during exercise. The increase was higher during LI compared to HI (Cmax: 201.8 nmol/L after 25 min vs. Cmax: 125.8 nmol/L after 25 min). After the cessation of exercise, vitamin B_6_ concentration diminished significantly reaching baseline again 19 h post-exercise.

The correlation analysis among the serum concentration of tHcy and the different vitamins analyzed showed a large variability and no relevant tendency was observed.

Energy, macronutrient, folate, vitamin B_12_, and vitamin B_6_ intake during the experimental trial days, compared to the RDA and AMDR [26], [27], are shown in Table 3. The dietary intake of the volunteers was in accordance with the proposed targets for energy (% of target intake: 91.9%), macronutrients (CHO: 103.1%; Proteins: 85.3%; Lipids: 72.7%), and vitamins (Folates: 228.4%; Vitamin B_12_∶ 686.0%; Vitamin B_6_∶ 420.0%).

**Table 3:** Nutritional intake of volunteers (n = 8) during the experimental trial days, target energy intake, Recommended Dietary Allowances (RDA) and Acceptable Macronutrient Distribution Range (AMDR).

	Intake	Intake targets^a^
Energy (MJ)	12.0 (11.0–12.2)	12.0–13.4
Carbohydrates (%E)	67.5 (64.2–69.8)	45–65
Lipids (%E)	19.0 (16.0–22.0)	20–35
Proteins (%E)	14.0 (13.0–14.8)	10–35
Folate (µg)	646.0 (177.0–683.0)	300
Vitamin B_12_ (µg)	22.7 (3.2–25.7)	1.4
Vitamin B_6_ (mg)	6.2 (1.8–6.5)	1.5

Data are presented as Median (Interquartile range).

a Intake targets: For Energy intake the energy requirements were calculated using the Harris-Benedict equation [24], multiplied by a physical activity factor (1.4), and with 400 kcal added to account for the energy expenditure during the exercise trial. For Macronutrients and vitamins, the Acceptable Macronutrient Distribution Range (AMDR) [27] and the Recommended Dietary Allowances (RDA) [26] were used, respectively.

%E: percent of energy intake.

No relevant tendency was observed in the correlation analysis between tHcy and the intake of folates, vitamin B_12_, and vitamin B_6_ intake in the different meals throughout the trial days.

## Discussion

This study constitutes a holistic approach to the kinetics and metabolism of tHcy, an independent risk factor for CVD, in response to acute exercise at different intensities in sedentary individuals. To our knowledge, this is the first investigation that shows data on the variation of tHcy during exercise, providing a complete perspective of the kinetics of this parameter. Understanding this response could be relevant in terms of further informing healthy exercise recommendations.

An interesting finding in the present study is the observation that in response to an acute bout of exercise tHcy increases and Cmax occurs during exercise. From this point onwards, tHcy declines until the cessation of exercise. Thus, the response of tHcy to acute exercise is not linear, but biphasic, as evidenced by an initial increase and subsequent decrease, although the basal concentration is not recovered until 19 h post-exercise. The previous studies that have evaluated the impact on tHcy of an acute bout of exercise have not accounted for the variations during exercise, so they can only observe a linear relationship between pre and post-exercise tHcy. Furthermore, contradictory and inconclusive results were obtained, since some of them found acute exercise to increase tHcy, while others described a decrease in this parameter, and others found no effect at all [9], [11], [13], [32], [33], [34], [35]. Therefore, the differences in the values measured after exercise by the variety of authors could be related to differences in the timing of post-exercise sample collection, which may in fact represent different periods in the recovery phase. Furthermore, we have observed that Cmax coincided with a particular quantity of energy expended, irrespective of exercise intensity, but not of the duration of exercise.

Consequently our results show that post-exercise tHcy depends on the timing of post-exercise sample collection and on the total energy expenditure during the exercise trial, which could partially explain the heterogeneity in the results obtained in previous studies.

This observation could also explain in part the higher resting tHcy observed in physically active versus sedentary people [31], [36], [37]. In these studies the time elapsed after the last training session prior the blood sample collection was not specified. Thus, the higher basal tHcy reported in physically active people may be through the repeated, but transient, increase during each successive exercise bout. This could determine a state of permanent postexercise recovery, as observed for other plasma biomarkers in response to exercise [38].

Nevertheless, a high interindividual variability in the kinetics of tHcy were observed (Figure 2), so it would be interesting to confirm these findings in a larger sample.

**Figure 2:** Distribution of serum homocysteine concentration values in every sampling point at low and high intensity isocaloric exercise trials. Open bars, Low intensity exercise (40% VO_2peak_); Grey bars, High intensity exercise (80% VO_2peak_). Open dots represent outliers. *Significant differences in high intensity exercise (*P*<0.05) between pre0 vs. exer10, exer20, exer30, and post0. †Significant differences in high intensity exercise (*P*<0.05) between post19 vs. exer10, 20, 30, post0, and post 3. pre4: Blood sample 4 h before exercise; pre0: Blood sample immediately before exercise; exer10: Blood sample 10 min during exercise; exer20: Blood sample 20 min during exercise; exer30: Blood sample 30 min during exercise; exer45: Blood sample 45 min during exercise; exer60: Blood sample 60 min during exercise; post0: Blood sample immediately after exercise; post3: Blood sample 3 h after exercise; post19: Blood sample 19 h after exercise.

In the fasting state tHcy normally ranges from 5 to 15 µmol/L [39]. Thus, hyperhomocysteinemia has been defined as concentrations >15 µmol/L [5], [30]. We have found no values of hyperhomocysteinemia all over the exercise trials, irrespective of the intensity. However, this does not mean that the transient increase observed in tHcy is lacking of physiological relevance. A recent meta-analysis have found a 16% higher risk of ischemic heart disease in TT than CC for an average tHcy difference of 1.9 µmol/L [40]. This value coincides with the average increase in tHcy observed in our study in response to HI exercise (pre0 vs. Cmax). However, the increment in CVD risk reported by Wald et al. (2011) refers to a sustained elevation in tHcy throughout the lifespan, while our observation refers to an acute transient increase. Moderate acute elevations of tHcy through oral methionine load, also alter endothelial function in healthy adult humans [41], although it may be that the physiopathological consequences on CVD are different.

Several mechanisms have been proposed to explain the increase in tHcy post-exercise, when observed. Venta et al. (2009) [35] suggested that it is related to the transient reduction in renal blood flow and filtration that occurs after exercise. Other authors have proposed that the role of homocysteine as intermediate in amino acid synthesis after exercise induced muscle tissue damage, could also explain this increase [34], [36]. Unfortunately, neither mechanism explains the lack of a linear relationship between pre and post-exercise tHcy, or the decline during exercise at a time when the stimulus of exercise persists.

An alternative hypothesis is that the clearance observed for tHcy during exercise could be related to energy metabolism and substrate utilization. It is well known that substrate utilization changes during exercise in relation to the intensity and duration of the activity [42], and several authors have proposed a role of homocysteine in energy metabolism [31], [43]. As expected, we observed different substrate utilization profiles at LI vs. HI were observed throughout the exercise trials and at Tmax (RER, CHO and Lipid oxidation rate, and Total CHO and Lipid oxidized) [20]. However, no differences were found for Cmax at LI vs. HI, and the accumulated energy expenditure at Cmax was independent of the exercise intensity. Additionally, we have observed no correlation between tHcy and the serum concentration of vitamin B_6_ throughout the trials. In this sense, Crozier et al. (1994) [44], analyzing the kinetics of plasma PLP in response to exercise, postulate that the rise observed during exercise was not related to fuel provision.

Thus, in light of these results, no clear relationship can be established between tHcy kinetics during exercise and energy metabolism and fuel use, although further research is needed.

Furthermore, the predictors of tHcy may differ among populations according to their nutritional status. Folates, more than other B-vitamins, are essential to maintain safe homocysteine concentrations. An inverse relationship between tHcy and serum folate has been described, but only when the nutritional status for folic acid is adequate [45], [46], [47]. Despite the optimal folate status of the volunteers that took part in our study, an increase in tHcy was observed in response to exercise. So, in light of our results, adequate folate intake could be especially important for people that are seldom active, and who would be exposed to transient increases in tHcy.

In conclusion, acute exercise in young sedentary individuals transiently increases tHcy during exercise irrespective of the intensity, but does not result in hyperhomocysteinemia. Further research is needed to clarify the exact mechanism by which this increase occurs. Consequently, acute exercise, even of high intensity, has no negative effect on tHcy as an independent risk factor for CVD, when at least 400 kcal are spent during exercise and the nutritional status for folates is adequate. These results inform the response of a risk factor for CVD to acute exercise in sedentary people and are relevant for public health in terms of further informing healthy exercise recommendations.
